# Testing a bat fatality detection system at wind turbines

**DOI:** 10.1371/journal.pone.0334609

**Published:** 2025-11-07

**Authors:** Sara P. Weaver, Jon D. Ritter, Alexis M. Commiskey, Juan D. Garcia, Brogan P. Morton

**Affiliations:** 1 Natural Resources, Bowman Consulting, San Marcos, Texas, United States of America; 2 Wildlife Imaging Systems, Hinesburg, Vermont, United States of America; King Fahd University of Petroleum & Minerals, SAUDI ARABIA

## Abstract

To understand conditions associated with bat fatalities at wind turbines for informing reduction strategies, researchers began using thermal camera video monitoring with a field of view (FOV) focused on the rotor swept area (RSA) to detect fatalities. However, confidently detecting fatalities and correctly classifying when they occur in the RSA is difficult and relatively few have been documented when compared to the hours of recordings produced to date. We conducted the first proof-of-concept study to determine whether a ground-based thermal camera system focused below the RSA, combined with machine learning algorithms, could effectively track and detect bat fatalities at wind turbines. To determine camera success, we equipped two wind turbines in southern Texas each with two cameras and performed standard post-construction monitoring (PCM). We classified a total of 274,051 bat tracks, of which 189 were identified as potential bat fatalities by machine learning algorithms, while the remaining tracks corresponded to bats flying within the camera’s FOV. After manual review of 10-minute summary images of all recorded videos, 23 bat tracks identified by algorithms were also manually identified in video as possible fatalities that occurred in a camera’s field of view. These 23 tracks also aligned with a searcher discovered bat carcass in the detection space of the corresponding camera with an estimated time of death overlapping with a night of an identified track. Our findings demonstrate that the camera system, paired with our proprietary machine learning algorithm, can process thousands of hours of video to identify individual tracks as possible bat fatalities. We propose that the primary value of this system lies in its ability to automatically process many hours of video data and identify suspected bat fatality tracks which could direct human searchers to specific turbines in an effort to minimize manual searches, as well as its potential application in estimating offshore fatalities in settings where traditional search methods are not feasible.

## Introduction

Research on wind-turbine related bat fatalities has revealed higher bat activity, as well as fatality, during nights of lower wind speeds [1–3]. This knowledge led to blanket curtailment of wind turbines at night during periods of low wind speed as the primary bat fatality reduction strategy recommended by regulators and in practice today [4–6]. While blanket curtailment can significantly reduce bat fatalities [4,5,7], this method results in power production losses for wind energy facilities [5,8,9]. In addition, research indicates bats are only active around a curtailed turbine for a fraction of the night [10,11] resulting in power production loss when blanket curtailment is implemented but bats are not present. It is therefore of interest to find ways to reduce bat fatalities that lessen these power losses by identifying other conditions influencing mortality rates to inform when turbines should be curtailed, a strategy often termed smart curtailment [12–14]. This could be accomplished through a better understanding of site-specific bat behavior at wind turbines by answering the questions: when and under what conditions (e.g., meteorological, spatial, temporal, etc.) is bat fatality most often occurring at wind turbines? Answering this question will inform on the causal mechanisms of collision risk and result in improvements to smart curtailment strategies.

To understand conditions associated with bat fatality at wind turbines, researchers began using thermal camera video monitoring with a field of view (FOV) in the rotor swept area (RSA) [15–17]. While these studies were conducted to monitor bat behavior around and interactions with wind turbines, they noted occurrences in which it appeared a bat was struck by a moving blade. However, confidently detecting a fatality and correctly classifying when it occurs in the RSA is difficult for a variety of reasons, leaving researchers to be uncertain if a fatality has occurred [15,16]. The distance from the camera and size of bats compared to turbine blades is part of the difficulty, but bats can also have close encounters or even what appears to be a strike but recover and fly out of the FOV leaving researchers uncertain of the outcome. Confidence can improve if video monitoring is paired with post-construction fatality monitoring (PCM) and carcasses are found the day following a suspected wind-turbine blade collision event, however finding carcasses during PCM can also be difficult [18,19]. Thus, various wind energy facilities now use bat acoustic activity monitored with acoustic detectors at wind turbine as a measure of bat exposure and a proxy for bat fatality risk [10,20]. This method allows researchers to document the precise spatial, temporal, and meteorological conditions occurring when bats are active around a wind turbine which can then inform smart curtailment by assuming activity is related to risk [12,20].

While more cost-effective than video monitoring, acoustics have many limitations, including detection range due to sound attenuation (more so for higher frequency-calling bats) and they do not always record bats even when they are present at wind turbines [21,22]. In fact, recent research indicates hoary bats (*Lasiurus cinereus*), including Hawaiian hoary bats (*L. cinereus semotus*), sometimes produce quieter calls during flight possibly to reduce competition [21,23]. Gorresen et al. [21] reported that on average only one in three visual bat detections using nocturnal video monitoring technology within a night had an accompanying acoustic call detection. Additionally, acoustic recordings cannot determine the number of bats present, as 100 call files could represent 100 bats each producing a single call, a single bat calling 100 times, or any variation in between. This provides evidence that nocturnal video monitoring may still offer a more comprehensive analysis of bat activity and fatality at wind turbines and the conditions under which they occur.

Focusing a camera’s FOV on the RSA to determine the timing of collision events may not be the most effective approach, as previously discussed. If a blade strike results in fatality, the bat’s expected trajectory would involve falling to the ground. This descent might be more readily detected by cameras focused below the RSA. To our knowledge, this area around wind turbines has not been studied using thermal cameras for bat fatalities. Therefore, we questioned whether a thermal camera system focused below the RSA could provide a more reliable detection of falling objects, including bats. Our objective was to conduct a proof-of-concept study to test a thermal camera system’s capability of accurately detecting wildlife fatalities, with a focus on bats, at wind turbines by concentrating the FOV below the RSA. If successful, this approach could lead to improved site-level strategies to mitigate risks for bats and provide a method for detecting wildlife fatalities at offshore wind turbines where standard observer search methods are not feasible.

## Materials and methods

### Study site

Our study site was the Reloj del Sol Wind Farm (RDS) located in Zapata County, Texas. RDS became operational in early 2022 with a total of 63 Nordex Acciona turbines (17 3.0 megawatt [MW]; 6 3.3 MW; 40 3.5 MW) with a 132 m rotor diameter for a generating capacity of approximately 200 MW. Wind turbines were feathered up to the manufacturer cut-in speed of 3.0 m/s during our study.

The project area at RDS is approximately 8,325 hectares located northeast of San Ygnacio, Texas, and is within the Texas-Tamaulipan Thornscrub Level IV ecoregion within the South Texas Plains Level III ecoregion [24]. The Texas-Tamaulipan Thornscrub ecoregion physiography is described as lightly to moderately dissected irregular plains. The mean annual precipitation ranges from 508 to 660 mm and land use and cover are primarily shrub/scrub, pastureland, ranching, hunting leases, and some oil and gas production [24].

This study was carried out in strict accordance with the guidelines set forth by the American Society of Mammalogists and Texas Parks and Wildlife Department permit number SPR-1120–189.

### Camera deployment and study design

We deployed a thermal camera system mounted at ground level providing a view of the airspace around a wind turbine just above ground-level and below the RSA at two 3.5 MW wind turbines (T114 and T156) at RDS. The systems were operational nightly from July 15^th^ to October 31^st^, 2022. We pointed each camera approximately 15 degrees above the horizon and powered it with a solar panel and battery storage power system. The FOV included part of the turbine tower on the left side and sky as a reference point. We programmed the cameras to operate from at least 2 hours before sunset to 2 hours after sunrise of the longest night during the study, occurring October 31st.

At each wind turbine, we deployed two Axis Q1952-E thermal cameras with a 35 mm lens on tripods approximately 75 m from the turbine looking back towards it, one on the northside facing south and one to the southside facing north, such that they covered an approximate 50-meter by 100-meter rectangular area within the search plot around the turbine (Fig 1). The search plots encompassed the full FOV of each camera and additional areas outside the FOV to the east and west to adhere to study design for concurrent PCM efforts.

**Fig 1:** A model of the airspace monitored by the two Axis Q1952-E thermal cameras. Each thermal camera (red pins) was placed 75 meters away from the turbine and had a field of view (yellow volume) whose left edge includes the tower.

The wind turbines we selected were a subset of six full-plot turbines already under standard PCM for bat fatalities for due diligence purposes. To maximize sample sizes for this proof-of-concept study, we selected the two turbines with the highest number of bat carcasses discovered during PCM efforts leading up to deployment of the camera systems. However, three days after the study began, T156 was taken offline indefinitely due to blade integrity issues. Thus, we moved this system to T101 on July 27^th^. We selected T101, which was a 3.0 MW wind turbine, primarily because the search area was not truncated (as was the case for the other full plot turbines) and would allow for the full FOV of each camera to be searched and was the next highest on number of carcasses found to date.

### Post-construction fatality monitoring

Qualified biologists conducted standard bat carcass searches four consecutive days a week whenever possible at both turbines with cameras deployed [25]. We were unable to conduct daily searches for the duration of the study due to funding constraints. Individuals conducting carcass searches were unaware of when or where bat fatalities occurred because camera data were not processed and analyzed in real time, so there was no opportunity for searcher bias based on known fatalities from camera detections. While cameras operated seven days a week, weather occasionally caused delays in search efforts. Thus, some searches were conducted multiple days after a detected fatality by the cameras. We searched 100 m by 100 m square plots centered on the wind turbine which encompassed the FOV of the camera system plus additional areas to the east and west. We spaced transects 5 m apart within each full plot and observers searched 2.5 m on each side of the transect line. With the camera FOV being a subset of the full searched plot, we acknowledged that carcasses were likely to be found outside the expected FOV and the total carcass count was biased to only look at the fatalities we expected the cameras to find. Otherwise, the cameras in this proof-of-concept testing were likely to be penalized for missing fatalities that occurred outside their FOV. We compared bat carcasses discovered during searches with camera data to test the system’s ability to detect a carcass falling through the FOV.

### Video analysis

We calculated summary statistics for each camera system and wind turbine. A thermal camera night was considered a single camera recording for one night. We processed all videos using proprietary algorithms in the Python programming language to identify bat fatalities by detecting ‘tracks’ of associated detections. We used a background subtractor to automatically detect objects in the video stream. The algorithm detected all ‘new’ objects (e.g., bats, insects, birds) by dynamically modeling the image background, subtracting it from the incoming image, and determining which parts of the image deviated substantially. Those ‘different’ parts of each image are identified as detections. Using pixels from the area of each detection, the algorithm derived information about each object’s pixel location, area, width, length, and other distinguishing features. In addition to the quantitative outputs, a composite image that summarizes the detections found in every 5 minutes of video was created, providing a manual way to interpret the video.

Next, the algorithm connected detections into tracks, with each track representing a path followed by a single object through time. The algorithm required each connected detection within a track to be both spatially and temporally close (determined by proprietary coding) and can eliminate ‘noise’ (disconnected detections) in the dataset based on distance. Once tracks were generated, the algorithm quantified associated features, such as velocity and acceleration statistics, as well as the average size of the detections within the track. After tracks and features have been generated, the software saved them into a separate database.

Because bats are not the only objects that cameras could detect, we classified each track as a bat, insect, or other object using the associated features detailed above. To classify each track, a dataset was built by meticulously going through 10,000s of tracks and manually labeling each one as an object commonly seen in video (e.g., bat, bird, insect, blade, etc.) to create a labeled dataset. This manual training of the algorithm was a part of a Department of Energy Small Business Innovation Research grant (DE‐SC0021867). A model was then built based upon the labeled data to classify the remaining 100,000s of tracks. The model was built using features of the detections that can separate each track into its classified category.

We further classified each bat track as either activity or fatality based on the detection attributes. Since bat fatality is a rare event, to get enough training data for this model we created a physics-based model of a falling bat carcass and generated thousands of tracks to simulate a fatality. We were then able to supplement this synthetic data with the tracks we found through manual review of all composite images to be the fatalities used to create the final model. More than 7,000 hours of videos were collected, and we determined it was not feasible to watch and review all the videos. Instead, every composite image (more than 40,000) was reviewed manually to look for possible fatalities and to verify that the machine learning algorithm was not missing possible fatalities.

### Matching of PCM and video analysis data

We cross-referenced classified bat fatality tracks with searcher discovered carcasses with an adjustment for time of death if the carcass was not fresh. For example, if a carcass was estimated to be two to three days old, we would assign the fatality window as having potentially occurred two to three days prior for review of camera detections. We determined time of death using multiple factors, such as wing pliability, insect infestation, condition of the eyes, and smell. In addition, we had previous knowledge of desiccation rates in this region from field trial studies designed to accurately estimate time of death [25], reducing errors in time of death estimates. When the timestamp of a classified bat fatality track fell within the estimated fatality window of a searcher discovered carcass, we considered those to be a match.

We acknowledge that the temporal correlation between a classified bat fatality track and a searcher discovered carcass does not prove the two are definitively matched. It is possible the camera system detected a fatality that was not subsequently found by a searcher or a searcher found a carcass that was not detected by the camera system. We believe this will be a systemic issue faced during testing of fatality detection systems at operational wind turbines that rely on carcass recovery for verification. At the time of this proof-of-concept study, the system was not capable of providing real-time alerts, which in the future could allow for immediate search efforts for more reliable correlations. In the face of these limitations, we will consider the temporal correlations to be sufficient evidence of a match.

During video analysis, we unexpectedly discovered a high magnitude of bat flight activity in the FOV (Fig 2). Thus, we decided post hoc to quantify bat activity in addition to fatality. Each detection represented 1/30^th^ of a second (the length of time between video frames) of activity in the video FOV. Thus, we summed all detections of bats over a determined period and divided by 30 to create an activity metric. As an example, if there were 1,234 bat detections in a ten-minute period, that would represent 1,234/30 = 41.1 bat-seconds of activity. Since each detection had a time stamp with resolution to a fraction of a second, we were able to easily bin each detection into different time periods.

**Fig 2:** Bat activity tracks (yellow) below the rotor swept area classified by a proprietary machine learning algorithm during a 10-minute period at wind turbine T101 on August 12, 2022, at Reloj del Sol Wind Farm in Zapata County, Texas.

To quantify error, we sorted fatalities into the following three categories:

- *Matched Positives (MP)*: Fatalities that were both found by human searches and detected by the camera system.
- *Camera False Positive (CFP)*: Camera-detected fatalities that DO NOT have a matching searcher discovered fatality.
- *Camera Negative (CN)*: Searcher-discovered fatalities that DO NOT have a matching camera-detected fatality.

We acknowledge the inherent issue with using searcher-discovered fatalities as a baseline for comparison to camera detected fatalities because not all fatalities that occur around a turbine will be found by searchers due to carcass persistence and searcher efficiency [19,26]. This can also be true of camera-detected fatalities as the camera may not detect all bat activity around a wind turbine due to limited FOV and may misidentify a track. However, the latter can be reduced with human review of summary images to select videos for manual review. Human searchers represent one of the best available and realistic methods for testing at the proof-of-concept phase. Thus, we used the searcher-discovered fatalities to calculate a representative value for MP and CN, but we could not do the same for CFP because there was a possibility the system detected an actual fatality that was not found during searches. To provide for that possibility, we reported two CFP values, one based on a strict comparison to the searcher discovered fatalities and one based on manual review of the videos to determine if the prediction was potentially a fatality that was not found by searchers. We further investigated missed camera detections (CN) to determine if the root cause of the miss was due to poor imaging, the detection algorithm, or the classification algorithm. From these numbers we characterized three metrics for the camera system:

- *Matched detection rate*: The percentage of all fatalities found by human searchers and detected by the system. Equation: $\frac{MP}{MP+CN}*\text{1}\text{0}\text{0}$
- *Camera missed detection rate*: The percentage of all fatalities found by human searchers NOT detected by the system. Equation: $\frac{CN}{MP+CN}*\text{1}\text{0}\text{0}$
- *Camera false detection rate*: The percentage of all the camera detected fatalities that were NOT matched fatalities. Equation: $\frac{CFP}{MP+CFP}*\text{1}\text{0}\text{0}$

These equations are based on standard performance evaluation metrics in classification tasks [27,28]. While the application to camera-based bat fatality detection is unique to our study, the metric definitions follow conventional forms of sensitivity, false negative rate, and false discovery rate [29].

## Results

We completed a total of 51 searches at T101 and 57 searches at T114. We chose not to include data from T156 because blade integrity issues can cause inconsistent wind turbine operations and we were uncertain if the wind turbine was operational during the three nights of video recordings. We were only able to complete one search at T156 with no carcasses detected before it was taken offline, and thus we chose to not include these data in analyses. A total of 40 bat carcasses were found by searchers during our study, 34 at T101 and six at T114. This included all carcasses discovered during standard PCM, regardless of location relative to camera FOV. The most discovered bat species was the Brazilian free-tailed bat (*Tadarida brasiliensis*).

The cameras recorded a combined total of 200 thermal camera nights at T101 across the two systems and 216 thermal camera nights at T114, resulting in 416 thermal camera nights across all four cameras. The systems operated as expected, with no equipment malfunctions reported during the study. However, a failure occurred at the southern camera system at T101 due to human error, rendering it non-operational from August 12 to August 28. As a result, data from these nights were unavailable for that camera.

We classified a total of 274,051 bat tracks, of which 189 were identified by machine learning algorithms as potential fatalities, while the remaining tracks corresponded to bats flying within the camera’s FOV. For each of the 189 tracks, the video was then manually reviewed to determine if the track should be further compared to the carcasses found. This required judgement from a human reviewer to determine if the track was likely a bat and if it was falling toward the ground versus still flying. Without ground truth data representing exactly when and where the fatality happened, manually watching the video represented the best option to correlate a possible fatality track happening during the window of expected fatality to a found carcass.

Of the 40 carcasses discovered by human searchers, we assumed 30 occurred within the camera system’s FOV based on their GPS locations at the time of discovery (e.g., within the 50 m x 100 m area within the search plot) and included them in further analysis. The 10 excluded occurred outside the camera FOV but were discovered due to the concurrent PCM searches which occurred in a larger area. Three fatalities were discovered by searchers within the camera’s FOV but were not detected by the cameras during our initial human review or by the machine learning algorithm. Additionally, two carcasses were found at T101 that had been missed due to the camera being offline, and two others were missed due to occlusion by the tower (discovered in the shadow of the turbine tower of the corresponding camera, but inside the 50-meter by 100-meter rectangle we expected the camera to find fatalities). In total, 23 carcasses were discovered by searchers and were correlated to a track detected by the camera system in the same area of the discovered carcass and considered MPs. A summary of this data is presented in Table 1.

**Table 1:** Summary of bat carcasses discovered and tracks detected.

Total Carcasses Discovered	40
Carcasses Discovered Outside the FOV of the Cameras	10
**Carcasses Discovered within the FOV of the Cameras**	30
Tracks Missed by Occlusion	2
Tracks Missed When System was Non-operational	2
Tracks Not Detected (CN)	3
**Tracks Detected by the System (MP)**	23

One additional fatality track was detected by the cameras and deemed highly likely to be a fatality but was not found by searchers. However, we could not confirm this fatality. Fig 3 provides an example of a fatality detected by the cameras that was also detected by searchers. Furthermore, the cameras classified 165 potential fatalities that were later determined to be CFPs. If the excluded fatality track detected by the cameras but not found by searchers was included, then there were 166 CFPs. The success metrics derived from these data are presented in Table 2. Thermal cameras also detected bat activity below the RSA at both wind turbines, with peak activity occurring during a single one-hour interval at T101 on October 20 and at T114 on October 28. The night with the highest overall bat activity across both turbines was October 28 (Figs 4 and 5).

**Table 2:** Summary of calculated success metrics for thermal camera detection of bat fatalities during at Reloj del Sol Wind Farm, July 15–October 31, 2022.

Matched Positives	Camera False Positives^a^	Camera False Positives^b^	Camera Negatives	Matched Detection Rate	Camera False Detection Rate^a^	Camera False Detection Rate^b^	Camera Missed Detection Rate
23	165	166	3	88.5%	87.8%	87.8%	11.5%

^a^Does not include the camera detected fatality track without a corresponding searcher discovered carcass.

^b^Includes the camera detected fatality track without a corresponding searcher discovered carcass.

**Fig 3:** Bat activity tracks (yellow) and a bat fatality track (red) classified by proprietary machine learning algorithms during a 10-minute period at wind turbine T101 on August 12, 2022, at Reloj del Sol Wind Farm in Zapata County, Texas.

**Fig 4:** Seconds of bat activity binned by hour across a night at wind turbine 101 during the study period at Reloj del Sol Wind Farm in Zapata County, Texas.

**Fig 5:** Seconds of bat activity binned by hour across a night at wind turbine 114 during the study period at Reloj del Sol Wind Farm in Zapata County, Texas.

## Discussion

We conducted the first proof-of-concept study to evaluate whether a ground-based thermal camera system focused below the RSA could effectively track and detect bat fatalities at wind turbines. Our findings demonstrate that the system, combined with our proprietary machine learning algorithm, can process thousands of hours of video to identify individual tracks as possible fatalities. With further testing and refinement, this system could provide an additional method for identifying the moment of a bat fatality and the conditions under which they occur, which could in turn assist in refining smart curtailment algorithms. Additionally, this system could be used at offshore wind turbines where traditional fatality monitoring methods are not feasible.

To our knowledge, only two other studies have evaluated thermal camera technology for detection of wildlife fatalities, including bats, occurring at wind turbines [30,31]. The B-finder system employs ring-shaped arrays of thermal cameras positioned at three vertical levels around the wind turbine tower to capture a full 360° view for detecting falling objects. Similar to our system, it focuses on the ability to detect objects falling to the ground. However, unlike our system, it is not ground-based making access for system checks and maintenance more difficult, and requires at least 48 thermal cameras, resulting in high equipment costs. Additionally, to our knowledge, no peer-reviewed results have been published. Happ et al. [31] evaluated a thermal camera system designed to be mounted in a turbine nacelle, with its FOV directed towards the ground, to detect bat fatalities by identifying pixel changes before and after a carcass landed. Although their FOV included areas below the RSA, the system was also not ground-based, requiring holes to be drilled into a wind turbine nacelle making it less cost-effective, and relied on different metrics to detect fatalities making direct comparisons of efficacy difficult. Like our approach, however, it faced challenges with camera false positives [31]. Similarly, our system’s initial classification model misclassified an unrealistic number of tracks. We determined this by comparing to the per turbine bat mortality rate corrected for bias and estimated with GenEst [32] from concurrent PCM efforts (S. Weaver, personal communication, 2022), which if we sum for two wind turbines since we did not assess misclassification per turbine, is approximately 4 times larger and nearly 7 times larger than the highest and lowest estimated bat mortality rate based on 90% confidence intervals from concurrent PCM efforts. As detection algorithms and classification models evolve, we anticipate a substantial reduction in CFP, leading to improved system accuracy.

A key outcome of this research is verification that the technology can detect wildlife fatalities when focused below the RSA. The rate of CFP is still too high and requires the model to be improved before it can be used commercially. Once the technology matures, this capability could enable the development of more refined smart curtailment algorithms based on the specific conditions influencing fatalities, potentially increasing power production while still mitigating bat fatalities [12,14]. Additionally, we observed high bat activity below the wind turbine RSA—a significant finding, as deterrent technologies, and detection equipment for studying bat behavior have traditionally been focused on the RSA and nacelle of wind turbines [15,25]. Furthermore, as wind turbine RSAs grow larger and blade tips extend closer to the ground, understanding the full vertical profile of bat activity will be crucial for assessing whether these changes introduce additional risks to bats [33,34].

We are uncertain why three fatalities discovered by human searchers were not detected by the camera system (considered 3 CN). Most likely, the detection algorithms require further refinement to identify all fatality tracks within the camera’s FOV. In this proof-of-concept testing, not only were we testing the technology and system, but we were creating the models to classify all the data. As technology matures and the model becomes more accurate, we expect CNs to decrease. Another plausible explanation is that the locations where the bat carcasses were found may not represent where the fatalities initially occurred or where the bats originally fell. Not all bats discovered below wind turbines are immediately fatally injured [35–37]. If a bat was injured while flying near a turbine and fell to the ground but was not yet dead, it might have moved from that spot depending on the severity of the injury. This makes it challenging to determine where the strike occurred and whether the cameras should have detected it. Furthermore, factors such as partial scavenging and environmental conditions, including high winds and stormwater runoff, could displace carcasses from their original locations.

We recognize that future testing of this system will require further validation of the tracks seen and carcasses found. This study was not meant to be a statistically rigorous validation, but a test for a proof-of-concept system that can be fully validated with additional funding. To validate that the tracks are bat fatalities will likely require three-dimensional modeling paired with daily searches, or real-time triggers that could allow for near immediate search efforts. Unfortunately, because of the lack of other technologies that may detect falling carcasses, we will likely still have to assume carcasses found and classified fatality tracks from the same night are likely matching, instead of being able to prove they are. The lack of ground truth data will always handicap the validation of this system type but allowing these correlations to help refine the model will speed up development. That and focusing on designing a future system where these possible fatality tracks help human searchers a specific area of a specific turbine will create a feedback loop that should lead to improved results, in the long-term.

We utilized a two-camera system in this study to balance system complexity and cost against coverage area. While deploying a larger system with additional cameras and equipment could improve coverage [30] and detection of bat activity and fatalities, it would also significantly increase both capital and recurring expenses. Based on discussions with industry operators and original equipment manufacturers (OEMs), we believe such a system would be economically impractical for commercial implementation. The two-camera setup used in this study represents the maximum viable configuration for maintaining cost-effectiveness. Additionally, we caution against using this system as a replacement for human or dog-handler teams during PCM, as it cannot identify species, cannot account for bias in mortality estimation in its current stage of development, and has a limited FOV. Instead, we propose that the primary value of this system lies in its ability to automatically process many hours of video data down to individual tracks to one day, direct human searchers to specific turbines in an effort to minimize manual searches, as well as its potential application in estimating offshore fatalities in settings where traditional search methods are not feasible.
